# ‘Green’ synthesis of metals and their oxide nanoparticles: applications for environmental remediation

**DOI:** 10.1186/s12951-018-0408-4

**Published:** 2018-10-30

**Authors:** Jagpreet Singh, Tanushree Dutta, Ki-Hyun Kim, Mohit Rawat, Pallabi Samddar, Pawan Kumar

**Affiliations:** 1 Department of Nanotechnology, Sri Guru Granth Sahib World University, Fatehgarh Sahib, Punjab 140406 India; 2 Department of Chemical, Biological & Macromolecular Sciences, S. N. Bose National Centre for Basic Sciences, Block JD, Sector III, Salt Lake, Kolkata 700 098 India; 3 Department of Civil & Environmental Engineering, Hanyang University, Seoul, 04763 South Korea; 4 Department of Nano Science and Materials, Central University of Jammu, Jammu, J & K 180011 India

**Keywords:** Green synthesis, Metals, Metal oxide nanoparticles, Natural extracts

## Abstract

In materials science, “green” synthesis has gained extensive attention as a reliable, sustainable, and eco-friendly protocol for synthesizing a wide range of materials/nanomaterials including metal/metal oxides nanomaterials, hybrid materials, and bioinspired materials. As such, green synthesis is regarded as an important tool to reduce the destructive effects associated with the traditional methods of synthesis for nanoparticles commonly utilized in laboratory and industry. In this review, we summarized the fundamental processes and mechanisms of “green” synthesis approaches, especially for metal and metal oxide [e.g., gold (Au), silver (Ag), copper oxide (CuO), and zinc oxide (ZnO)] nanoparticles using natural extracts. Importantly, we explored the role of biological components, essential phytochemicals (e.g., flavonoids, alkaloids, terpenoids, amides, and aldehydes) as reducing agents and solvent systems. The stability/toxicity of nanoparticles and the associated surface engineering techniques for achieving biocompatibility are also discussed. Finally, we covered applications of such synthesized products to environmental remediation in terms of antimicrobial activity, catalytic activity, removal of pollutants dyes, and heavy metal ion sensing.

## Introduction

Over the last decade, novel synthesis approaches/methods for nanomaterials (such as metal nanoparticles, quantum dots (QDs), carbon nanotubes (CNTs), graphene, and their composites) have been an interesting area in nanoscience and technology [1–9]. To obtain nanomaterials of desired sizes, shape, and functionalities, two different fundamental principles of synthesis (i.e., top down and bottom up methods) have been investigated in the existing literature (Fig. 1). In the former, nanomaterials/nanoparticles are prepared through diverse range of synthesis approaches like lithographic techniques, ball milling, etching, and sputtering [10]. The use of a bottom up approach (in which nanoparticles are grown from simpler molecules) also includes many methods like chemical vapor deposition, sol–gel processes, spray pyrolysis, laser pyrolysis, and atomic/molecular condensation.

**Fig. 1:** Different synthesis approaches available for the preparation of metal nanoparticles

Interestingly, the morphological parameters of nanoparticles (e.g., size and shape) can be modulated by varying the concentrations of chemicals and reaction conditions (e.g., temperature and pH). Nevertheless, if these synthesized nanomaterials are subject to the actual/specific applications, then they can suffer from the following limitation or challenges: (i) stability in hostile environment, (ii) lack of understanding in fundamental mechanism and modeling factors, (iii) bioaccumulation/toxicity features, (iv) expansive analysis requirements, (v) need for skilled operators, (vi) problem in devices assembling and structures, and (vii) recycle/reuse/regeneration. In true world, it is desirable that the properties, behavior, and types of nanomaterials should be improved to meet the aforementioned points. On the other hand, these limitations are opening new and great opportunities in this emerging field of research.

To counter those limitations, a new era of ‘green synthesis’ approaches/methods is gaining great attention in current research and development on materials science and technology. Basically, green synthesis of materials/nanomaterials, produced through regulation, control, clean up, and remediation process, will directly help uplift their environmental friendliness. Some basic principles of “green synthesis” can thus be explained by several components like prevention/minimization of waste, reduction of derivatives/pollution, and the use of safer (or non-toxic) solvent/auxiliaries as well as renewable feedstock.

‘Green synthesis’ are required to avoid the production of unwanted or harmful by-products through the build-up of reliable, sustainable, and eco-friendly synthesis procedures. The use of ideal solvent systems and natural resources (such as organic systems) is essential to achieve this goal. Green synthesis of metallic nanoparticles has been adopted to accommodate various biological materials (e.g., bacteria, fungi, algae, and plant extracts). Among the available green methods of synthesis for metal/metal oxide nanoparticles, utilization of plant extracts is a rather simple and easy process to produce nanoparticles at large scale relative to bacteria and/or fungi mediated synthesis. These products are known collectively as biogenic nanoparticles (Fig. 2).

**Fig. 2:** Key merits of green synthesis methods

Green synthesis methodologies based on biological precursors depend on various reaction parameters such as solvent, temperature, pressure, and pH conditions (acidic, basic, or neutral). For the synthesis of metal/metal oxide nanoparticles, plant biodiversity has been broadly considered due to the availability of effective phytochemicals in various plant extracts, especially in leaves such as ketones, aldehydes, flavones, amides, terpenoids, carboxylic acids, phenols, and ascorbic acids. These components are capable of reducing metal salts into metal nanoparticles [11]. The basic features of such nanomaterials have been investigated for use in biomedical diagnostics, antimicrobials, catalysis, molecular sensing, optical imaging, and labelling of biological systems [12].

Here, we summarized the current state of research on the green synthesis of metal/metal oxide nanoparticles with their advantages over chemical synthesis methods. In addition, we also discussed the role of solvent systems (synthetic materials), various biological (natural extracts) components (like bacteria, algae, fungi, and plant extracts) with their advantages over other conventional components/solvents. The main aim of this literature study is to provide detailed mechanisms for green synthesis and their real world environmental remediation applications. Overall, our goal is to systematically describe “green” synthesis procedures and their related components that will benefit researchers involved in this emerging field while serving as a useful guide for readers with a general interest in this topic.

## Biological components for “green” synthesis

Innumerable physical and chemical synthesis approaches require high radiation, highly toxic reductants, and stabilizing agents, which can cause pernicious effects to both humans and marine life. In contrast, green synthesis of metallic nanoparticles is a one pot or single step eco-friendly bio-reduction method that requires relatively low energy to initiate the reaction. This reduction method is also cost efficient [13–19].

### Bacteria

Bacterial species have been widely utilized for commercial biotechnological applications such as bioremediation, genetic engineering, and bioleaching [20]. Bacteria possess the ability to reduce metal ions and are momentous candidates in nanoparticles preparation [21]. For the preparation of metallic and other novel nanoparticles, a variety of bacterial species are utilized. Prokaryotic bacteria and actinomycetes have been broadly employed for synthesizing metal/metal oxide nanoparticles.

The bacterial synthesis of nanoparticles has been adopted due to the relative ease of manipulating the bacteria [22]. Some examples of bacterial strains that have been extensively exploited for the synthesis of bioreduced silver nanoparticles with distinct size/shape morphologies include: *Escherichia coli*, *Lactobacillus casei*, *Bacillus cereus*, *Aeromonas* sp. SH10 *Phaeocystis antarctica*, *Pseudomonas proteolytica*, *Bacillus amyloliquefaciens*, *Bacillus indicus*, *Bacillus cecembensis*, *Enterobacter cloacae*, *Geobacter* spp., *Arthrobacter gangotriensis*, *Corynebacterium* sp. SH09, and *Shewanella oneidensis*. Likewise, for the preparation of gold nanoparticles, several bacterial species (such as *Bacillus megaterium* D01, *Desulfovibrio desulfuricans*, *E. coli* DH5a, *Bacillus subtilis* 168, *Shewanella alga*, *Rhodopseudomonas capsulate*, and *Plectonema boryanum* UTEX 485) have been extensively used. Information on the size, morphology, and applications of various nanoparticles is summarized in Table 1.

**Table 1:** Examples of metallic nanoparticles prepared in ILs by a chemical reduction method

S. no.	Metal NPs	Metal salt	Reducing agent	Ionic liquid	Size (nm)	References
1	Ag	AgBF_4_	H_2_, 85 °C, 4 atm BIm as scavenger	[BMIm][BF_4_] [BMIm][PF_6_]	0.8–2.8 1.3–4.4	[148]
2	Ag	AgBF_4_	H_2_	[BMIm][BF_4_] [BMpy][TfO]	~ 9 (DLS) ~ 11 (DLS)	[149]
3	Ag	AgBF_4_	[BMIm][BH_4_]	[BMIm][BF_4_] purified and H_2_O	0.8–4.4 4.0 0.9–4.5	[47]
4	Ag	AgNO_3_	Tween 85	[BMIm][PF_6_]	3–10	[150]
5	Au	HAuCl_4_	Ascorbic acid	[BMIm] [C_12_H_25_OSO_3]_ (lauryl sulfate)	20–50	[151]
6	Au	HAuCl_4_	NaBH_4_	[ShexMIm][Cl]	5	[152]
7	Au	HAuCl_4_	NaBH_4_	[BMIm][BF_4_] in a microfluidic reactor	0.5–4	[153]
8	Au	HAuCl_4_-3H_2_O	Glycerol	[EMIm][TfO], [EMIm][MeSO_3_]	5–7 low temp. 5–7 aggregate at higher temp.	[154]
9	HAuBr_4_		Me_2_NCHO (DMF)	[Me_2_NH_2_][Me_2_NCO_2_] with small amounts of DMF	2–4	[155]
10	Cu	Cu(OAc)_2_-H_2_O	H_2_NNH_2_-H_2_O (hydrazine hydrate)	[BMIm][BF_4_]	80–130	[156]

### Fungi

Fungi-mediated biosynthesis of metal/metal oxide nanoparticles is also a very efficient process for the generation of monodispersed nanoparticles with well-defined morphologies. They act as better biological agents for the preparation of metal and metal oxide nanoparticles, due to the presence of a variety of intracellular enzyme [23]. Competent fungi can synthesize larger amounts of nanoparticles compared to bacteria [24]. Moreover, fungi have many merits over other organisms due to the presence of enzymes/proteins/reducing components on their cell surfaces [25]. The probable mechanism for the formation of the metallic nanoparticles is enzymatic reduction (reductase) in the cell wall or inside the fungal cell. Many fungal species are used to synthesize metal/metal oxide nanoparticles like silver, gold, titanium dioxide and zinc oxide, as discussed in Table 1.

### Yeast

Yeasts are single-celled microorganisms present in eukaryotic cells. A total of 1500 yeast species have been identified [26]. Successful synthesis of nanoparticles/nanomaterials via yeast has been reported by numerous research groups. The biosynthesis of silver and gold nanoparticles by a silver-tolerant yeast strain and *Saccharomyces cerevisiae* broth has been reported. Many diverse species are employed for the preparation of innumerable metallic nanoparticles, as discussed in Table 1.

### Plants

Plants have the potential to accumulate certain amounts of heavy metals in their diverse parts. Consequently, biosynthesis techniques employing plant extracts have gained increased consideration as a simple, efficient, cost effective and feasible methods as well as an excellent alternative means to conventional preparation methods for nanoparticle production. There are various plants that can be utilized to reduce and stabilize the metallic nanoparticles in “one-pot” synthesis process. Many researchers have employed green synthesis process for preparation of metal/metal oxide nanoparticles via plant leaf extracts to further explore their various applications.

Plants have biomolecules (like carbohydrates, proteins, and coenzyme) with exemplary potential to reduce metal salt into nanoparticles. Like other biosynthesis processes, gold and silver metal nanoparticles were first investigated in plant extract-assisted synthesis. Various plants [including aloe vera (*Aloe barbadensis* Miller), Oat (*Avena sativa*), alfalfa (*Medicago sativa*), Tulsi (*Osimum sanctum*), Lemon (*Citrus limon*), Neem (*Azadirachta indica*), Coriander (*Coriandrum sativum*), Mustard (*Brassica juncea*) and lemon grass (*Cymbopogon flexuosus*)] have been utilized to synthesize silver nanoparticles and gold nanoparticles, as listed in Table 2. The major part of this type of research has explored the ex vivo synthesis of nanoparticles, while metallic nanoparticles can be formed in living plants (in vivo) by reducing metal salt ions absorbed as soluble salts. The in vivo synthesis of nanoparticles like zinc, nickel, cobalt, and copper was also observed in mustard (*Brassica juncea*), alfalfa (*Medicago sativa*), and sunflower (*Helianthus annuus*) [27]. Also, ZnO nanoparticles have been prepared with a great variety of plant leaf extracts such as coriander (*Coriandrum sativum*) [28], crown flower (*Calotropis gigantean*) [29], copper leaf (*Acalypha indica*) [30], China rose (*Hibiscus rosa*-*sinensis*) [31], Green Tea (*Camellia sinensis*) [32], and aloe leaf broth extract (*Aloe barbadensis* Miller) [33]. Readers can refer to the work of Iravani [34] for a comprehensive overview of plant materials utilized for the biosynthesis of nanoparticles.

**Table 2:** Synthesis of metallic NPs from various biological species

Sr. no.	Species	Nanoparticles	Size (nm)	Morphology	Application	References
*Bacteria*						
1	*Bacillus cereus*	Silver	20–40	Spherical	Antibacterial activity against *Escherichia coli*, *Pseudomonas aeruginosa*, *Staphylococcus aureus*, *Salmonella typhi*, and *Klebsiella pneumonia* bacteria	[157]
2	*Pseudomonas proteolytica*, *Bacillus cecembensis*	Silver	6–13	Spherical	Antibacterial activity against *A. kerguelensis*, *A. gangotriensis*, *B. indicus*, *P. antarctica*, *P. proteolytica*, and *E. coli*	[158]
3	*Lactobacillus casei*	Silver	20–50	Spherical	Drug delivery, cancer treatments, bio-labeling	[159]
4	*Klebsiella pneumonia*, *Escherichia coli*, *Enterobacter cloacae*	Silver	28–122	Spherical	Optical receptors, electrical batteries, antimicrobial	[79]
5	*Bacillus indicus*	Silver	–	–	Antimicrobial, catalysis	[160]
6	*Plectonema boryanum UTEX 485*	Gold	< 10–25	Cubic, octahedral	–	[161]
7	*Bacillus subtilis 168*	Gold	5–50	Hexagonal-octahedral	–	[162]
8	*Bacillus megaterium D01*	Gold	< 2.5	Spherical	Catalysis, biosensing	[163]
9	*Shewanella alga*	Gold	pH 7: 10–20 pH 2.5: 15–200 pH 2: 20	Triangular	–	[164]
10	*E. coli DH 5α*	Gold	8–25	Spherical	Direct electrochemistry of hemoglobin	[165]
11	*Desulfovvibrio desulfuricans*	Gold	20–50	Spherical	Catalysis	[166]
12	*Rhodopseudomonas capsulate*	Gold	10–20	Cancer hyperthermia	Triangular	[167]
13	*Magnetospirillum magnetotacticum*	Iron Oxide	47	–	Handle shaped cluster	[168]
14	*Aquaspirillum magnetotacticum*	Iron Oxide	40–50	Octahedral prism	–	[169]
15	*Shewanella oneidensis*	Uranium oxide	1–5	–	–	[170]
16	*Klebsiella aerogenes*	Cadmium sulfide	20–200	–	–	[171]
17	*E. coli*	Cadmium sulfide	2–5	Fluorescent labels	Wurtzite structures	[23]
*Fungus*						
1	*Rhizopus nigricans*	Silver	35–40	Round	Bactericidal, catalytic	[172]
2	*Verticillium*	Silver	21–25	Spherical	Catalysis	[173]
3	*Aspergillus fumigates*	Silver	5–25	Spherical	Coating for solar energy absorption and intercalation material for electrical batteries	[174]
4	*Phanerochaete chrysosporium*	Silver	50–200	Pyramidal	Medical textiles for antimicrobial activity	[175]
5	*Aspergillus flavus*	Silver	1–8	–	Isotropic	[176]
6	*Aspergillus niger*	Silver	20	Spherical	Antibacterial agent	[177]
7	*Fusarium semitectum*	Silver	10–60	Crystalline spherical	Biolabelling	[178]
8	*Cladosporium cladosporioides*	Silver	10–100	Spherical	–	[179]
9	*Cariolus versicolor*	Silver	25–75	Spherical	Water-soluble metallic catalysts, labels for living cells and tissues	[180]
10	*Fusarium solani*	Silver	5–35	Spherical	Biolabeling, sensors, drug delivery	[181]
11	*Penicillium brecompactum*	Silver	23–105	Crystalline spherical	Antimicrobial agent	[182]
12	*Penicillium fellutanum*	Silver	5–25	Spherical	Thin film and surface coating	[183]
13	*Phoma glomerata*	Silver	60–80	Spherical	Antimicrobial agent	[184]
14	*Alternata alternate*	Silver	20–60	spherical	Antifungal agent	[185]
15	*Trichoderma viride*	Silver	5–40	Spherical	Antimicrobial agent	[186]
16	*Verticillium luteoalbum*	Gold	< 10	Triangular, hexagonal	Optics, sensor, coatings	[20]
17	*Rhizopus stolonifer*	Silver, Gold	25–30, 1–5	Spherical	–	[187]
18	*Trichothecium* sp.	Gold	10–25	Spherical, rod-like and triangular	–	[188]
19	*Fusarium oxysporum*	Gold-silver alloy	8–14	Spherical	Biomedical field	[189]
20	*Aspergillus terreus*	Zinc oxide	8	Spherical	Catalysis, biosensing, drug delivery, molecular diagnostics, solar cell, optoelectronics, cell labeling, and imaging	[190]
21	*Aspergillus flavus* TFR7	Titanium dioxide	12–15	Spherical	Plant nutrient fertilizer	[191]
*Yeast*						
1	MKY3	Silver	2–5	Hexagonal	Coatings for solar energy absorption and intercalation material for electrical batteries	[192]
2	*Saccharimyces cerevisae* broth	Gold, silver	4–15	Spherical	Catalysis	[193]

## Solvent system-based “green” synthesis

Solvent systems are a fundamental component in the synthesis process, whether it is “green” synthesis or not. Water is always considered an ideal and suitable solvent system for synthesis processes. According to Sheldon, “the best solvent is no solvent, and if a solvent is desirable then water is ideal” [35]. Water is the cheapest and most commonly accessible solvent on earth. Since the advent of nanoscience and nanotechnology, the use of water as a solvent for the synthesis of various nanoparticles has been carried out. For instance, synthesized Au and Ag nanoparticles at room temperature using gallic acid, a bifunctional molecule, in an aqueous medium [36]. Gold nanoparticles were produced via a laser ablation technique in an aqueous solution. The oxygen present in the water leads to partial oxidation of the synthesized gold nanoparticles, which finally enhanced its chemical reactivity and had a great impact on its growth [37].

In the literature, “green” synthesis consists of two major routes:

- Wherein water is used as a solvent system.
- Wherein a natural source/extract is utilized as the main component.

Both of these routes have been covered in the coming section according to the present literature. Hopefully, our efforts will help researchers gain a better knowledge of ‘green’ synthesis methods, the role of toxic/non-toxic solvents (or components), and renewable resources derived from natural sources. Ionic and supercritical liquids are one of the best examples in this emerging area. Ionic liquids (ILs) are composed of ions that have melting points below 100 °C. Ionic liquids are also acknowledged as “room temperature ionic liquids.” Several metal nanoparticles (e.g., Au, Ag, Al, Te, Ru, Ir, and Pt) have been synthesized in ionic liquids [38–41]. The process of nanoparticle synthesis is simplified since the ionic liquid can serve as both a reductant and a protective agent.

ILs can be hydrophilic or hydrophobic depending on the nature of the cations and anions. For example, 1-butyl-3-methyl imidazolium (Bmim) hexafluorophosphate (PF6) is hydrophobic, whereas its tetrafluoroborate (BF4) analogue is hydrophilic. Since both species are ionic in nature, they can act as catalysts [40, 42–45]. Bussamara et al. have performed a comparative study by controlling the synthesis of manganese oxide (Mn_3_O_4_) nanoparticles using imidazolium ionic liquids and oleylamine (a conventional solvent). They found that smaller sized nanoparticles (9.9 ± 1.8 nm) were formed with better dispersity in ionic liquids than in the oleylamine solvent (12.1 ± 3.0 nm) [46]. Lazarus et al. synthesized silver nanoparticles in an ionic liquid (BmimBF4). The synthesized nanoparticles were in both smaller isotropic spherical and large-sized anisotropic hexagonal shaped forms [47]. An electrochemical method was employed for this purpose [48]. Ionic liquid was used in the electrolytic reaction as a substitute for water without mechanical stirring. For the first time, Kim et al. developed a one-phase preparation technique for gold (Au) and platinum (Pt) nanoparticles by means of thiol-functionalized ionic liquids (TFILs). TFILs acted as a stabilizing agent to produce crystalline structures with small sizes [49]. Dupont et al. used 1-n-butyl-3-methylimidazolium hexafluorophosphate (which is room temperature ionic liquid) for synthesizing Ir(0) nanoparticles by Ir(I) reduction. The average size of synthesized nanoparticles was ~ 2 nm. Interestingly, the ionic liquid medium is impeccable for the production of recyclable biphasic catalytic systems for hydrogenation reactions [50].

The benefits of using ionic liquids instead of other solvents include the following. (a) Many metal catalysts, polar organic compounds, and gases are easily dissolved in ILs to support biocatalysts. (b) ILs have constructive thermal stabilities to operate in a broad temperature range. Most of these melt below room temperature and begin to decompose above 300 or 400 °C. As such, they allow a broader synthesis temperature range (e.g., three to four times) than that of water. (c) The solubility properties of IL can be modulated by modifying the cations and anions associated with them. (d) Unlike other polar solvents or alcohols, ILs are non-coordinating. However, they have polarities comparable to alcohol. (e) ILs do not evaporate into the environment like volatile solvents because they have no vapor pressure. (f) ILs have dual functionality because they have both cations and anions. The problems associated with the biodegradability of ionic liquids make them not acceptable for synthesis of metallic nanoparticles. To diminish these non-biodegradability issues, many new potentially benign ionic liquids are being developed with maximum biodegradation efficiency [51–54]. The innumerable ILs are used to synthesize various metallic nanoparticles as listed in Table 3.

**Table 3:** Green synthesis of metallic NPs from various plant extracts

Order	Plant origin	Nanoparticle	Size (nm)	Morphology	Applications	References
1	*Aloe barbadensis* Miller (Aloe vera)	Gold and silver	10–30	Spherical, triangular	Cancer hyperthermia, optical coatings	[194]
2	*Aloe barbadensis* Miller (Aloe vera)	Indium oxide	5–50	Spherical	Solar cells, gas sensors	[32]
3	*Acalypha indica*	Silver	20–30	Spherical	Antibacterial activity against water borne pathogens	[195]
4	Apiin extracted from henna leaves	Silver and gold	39	Spherical, triangular, and quasi-spherical	Hyperthermia of cancer cells and IR-absorbing optical coatings	[196]
5	*Avena sativa* (oat)	Gold	5–20 (pH 3 and 4),	Rod-shaped	–	[197]
6	*Azadirachta indica* (neem)	Gold, silver and silver-gold alloys	5–35 and 50–100	Spherical, triangular, hexagonal	Remediation of toxic metals	[198]
7	*Camellia sinensis* (black tea leaf extracts)	Gold and silver	20	Spherical, prism	Catalysts, sensors	[199]
8	*Brassica juncea* (mustard)	Silver	2–35	Spherical	–	[200]
9	*Cinnamomum camphora* (camphor tree)	Gold and silver	55–80	Triangular, spherical (Au), and quasi-spherical (Ag)	–	[85]
10	*Carica papaya* (papaya)	Silver	60–80	Spherical	–	[86]
11	*Citrus limon* (lemon)	Silver	< 50	Spherical, spheroidal	–	[201]
12	*Coriandrum sativum* (coriander)	Gold	6.75–57.91	Spherical, triangular, truncated triangular, decahedral	Drug delivery, tissue/tumor imaging, photothermal therapy	[202]
13	*Cymbopogon flexuosus* (lemongrass)	Gold	200–500	Spherical, triangular	Infrared-absorbing optical coatings	[203]
14	*Cycas sp.* (cycas)	Silver	2–6	Spherical	–	[204]
15	*Diospyros kaki* (persimmon)	bimetallic gold/silver	50–500	Cubic	–	[205]
16	*Emblica officinalis* (indian gooseberry)	Gold and silver	(10–20) and (15–25)	–	–	[206]
17	*Eucalyptus citriodora* (neelagiri)	Silver	20	Spherical	Antibacterial	[207]
18	*Eucalyptus hybrida* (safeda)	Silver	50–150	Crystalline, spherical	–	[208]
19	*Garcinia mangostana* (mangosteen)	Silver	35	Spherical	Antimicrobial activity against *E. coli* and *S. aureus*	[209]
20	*Gardenia jasminoides Ellis* (gardenia)	Palladium	3–5	–	Nanocatalysts for *p*-nitrotoluene hydrogenation	[210]
21	*Syzygium aromaticum* (clove buds)	Gold	5-100	Irregular	Detection and destruction of cancer cells	[211]
22	*Jatropha curcas* (seed extract)	Silver	15–50	Spherical	–	[212]
23	*Ludwigia adscendens* (ludwigia)	Silver	100–400	Spherical	–	[213]
24	*Medicago sativa* (alfalfa)	Gold	2–40	Irregular, tetrahedral, hexagonal platelet, decahedral, icosahedral	Labeling in structural biology, paints	[214–216]
25	*Mentha piperita* (peppermint)	Silver	5–30	Spherical	To kill microbes	[217]
26	*Medicago sativa* (alfalfa)	Iron oxide	2–10	Crystalline	Cancer hyperthermia, drug delivery	[218]
27	*Morus* (mulberry)	Silver	15–20	Spherical	Antimicrobial activity against *E. coli*, *B. subtilis*	[219]
27	*Nelumbo nucifera* (lotus)	Silver	25–80	Spherical, triangular, truncated triangular, decahedral	Larvicidal activity against malaria and filariasis vectors	[220]
28	*Ocimum sanctum* (tulsi; root extract)	Silver	10 ± 2 and 5 ± 1.5 nm	Spherical	Catalytic reduction	[221]
28	*Ocimum sanctum* (tulsi; leaf extract)	Gold and silver	30 and 10–20	Crystalline, hexagonal, triangular and spherical	Biolabeling, biosensor	[222]
29	*Pear fruit extract*	Gold	200–500	Triangular, hexagonal	Catalysis, biosensing	[223]
30	*Pelargonium roseum* (rose geranium)	Gold	2.5–27.5	Crystalline	–	[88]
31	*Psidium guajava* (guava)	Gold	25–30	Mostly spherical	–	[224]
32	*Sedum alfredii* Hance	Zinc oxide	53.7	Hexagonal wurtzite and pseudo-spherical	Nanoelectronics	[225]
33	*Tanacetum vulgare* (tansy fruit)	Gold and silver	11, 16	Triangular, spherical	Antibacterial, sensors	[226]
34	*Terminalia catappa* (almond)	Gold	10–35	Spherical	Biomedical field	[227]

Likewise, ordinary solvents can be converted into super critical fluids at temperatures and pressures above critical point. In the supercritical state, solvent properties such as density, thermal conductivity, and viscosity are significantly altered. Carbon dioxide is the most feasible super critical, non-hazardous, and inert fluid [55, 56]. Also, supercritical water can serve as a good solvent system for several reactions. As, water has critical temperature of 646 K and pressure of 22.1 MPa [57]. Silver and copper NPs can be synthesized in supercritical carbon dioxide [58]. Sue et al. suggested that decreasing the solubility of metal oxides around the critical point can lead to super saturation and the ultimate formation of nanoparticles [59]. Kim et al. synthesized tungsten oxide (WO_3_) and tungsten blue oxide nanoparticles by using sub- and supercritical water and methanol [60].

## Stability and toxicity of the nanoparticles

The environmental distribution and transport of released nanoparticles depend on their ability to make metastable aqueous suspensions or aerosols in environmental fluids. The stability of the nanoparticles in the environment can therefore be evaluated by estimating their propensity to aggregate or interact with the surrounding media. Aggregation is a time-dependent phenomena associated with the rate of particle collision while the stability of the suspension is largely determined by the size of the particles and affinity toward other environmental constituents. The “green” synthesis of AgNPs from tea leaf extraction was found to be stable after entering the aquatic environment [61]. Likewise, the stability of AgNPs (in aqueous medium) manufactured using plant extracts and plant metabolites was confirmed from the resulting material [62]. Surface complexation is also reported to affect the intrinsic stability of nanoparticles by regulating its colloidal stability. The nature and stability of nanoparticles were theoretically predicted through a mechanistic understanding of the surface complexation processes [63]. The colloidal stability (or rate of dissolution) of nanoparticles can be regulated by controlling the particle size and surface capping or through functionalization techniques [64, 65]).

Transformation of nanoparticles is an essential property to consider when assessing their environmental impact or toxicity. For instance, sulfurization of AgNPs greatly reduced their toxicity due to the lower solubility of silver sulfide [66]. For similar reasons, the use of biocompatible stabilizing agents (e.g., biodegradable polymers and copolymers) have opened up a “greener” avenue of nanomaterial surface engineering. Such techniques can impart remarkable stability, e.g., in situ synthesis of AuNPs capped with Korean red ginseng root [67]. Apart from surface chemistry, other key structural features determining the nanomaterial toxicity are the size, shape, and composition of the nanomaterials [68]. Toxicity analysis of AgNP synthesized using plant leaf extracts showed enhanced seed germination rates in the AgNP chemical treatment for activation than the corresponding control treatments [69]. However, the mechanism of such rate enhancement effects was not reported.

## Mechanism of “green” synthesis for metals and their oxide nanoparticles

### Microorganism-based mechanism

There are different mechanisms for the formation of nanoparticles using different microorganisms. First, metallic ions are captured on the surface or inside the microbial cells, and then these arrested metal ions are reduced into metal nanoparticles by the action of enzymes. Sneha et al. [70] described the mechanism of microorganism-assisted silver and gold nanoparticles formed via Verticillium sp. or algal biomass based on the following hypothesis. (a) First, the silver or gold ions were captured on the surface of fungal cells via electrostatic interactions between ions and negatively charged cell wall enzymes. (b) Then, silver or gold ions were bioreduced into silver or gold nuclei, which subsequently grew. The two key aspects in the biosynthesis of nanoparticles are NADH (nicotinamide adenine dinucleotide) and NADH-dependent nitrate reductase. Kalishwaralal et al. [71] demonstrated that the nitrate reductase was responsible for the production of bioreduced silver nanoparticles by *B. licheniformis*. Nonetheless, the bioreduction mechanisms associated with the production of metal salt ions and the resulting metallic nanoparticles formed by microorganisms remain unexplored.

### Plant leaf extract-based mechanism

For nanoparticle synthesis mediated by plant leaf extract, the extract is mixed with metal precursor solutions at different reaction conditions [72]. The parameters determining the conditions of the plant leaf extract (such as types of phytochemicals, phytochemical concentration, metal salt concentration, pH, and temperature) are admitted to control the rate of nanoparticle formation as well as their yield and stability [73]. The phytochemicals present in plant leaf extracts have uncanny potential to reduce metal ions in a much shorter time as compared to fungi and bacteria, which demands the longer incubation time [74]. Therefore, plant leaf extracts are considered to be an excellent and benign source for metal as well as metal oxide nanoparticle synthesis. Additionally, plant leaf extract play a dual role by acting as both reducing and stabilizing agents in nanoparticles synthesis process to facilitate nanoparticles synthesis [75]. The composition of the plant leaf extract is also an important factor in nanoparticle synthesis, for example different plants comprise varying concentration levels of phytochemicals [76, 77]. The main phytochemicals present in plants are flavones, terpenoids, sugars, ketones, aldehydes, carboxylic acids, and amides, which are responsible for bioreduction of nanoparticles [78].

Flavonoids contain various functional groups, which have an enhanced ability to reduce metal ions. The reactive hydrogen atom is released due to tautomeric transformations in flavonoids by which enol-form is converted into the keto-form. This process is realized by the reduction of metal ions into metal nanoparticles. In sweet basil (*Ocimum basilicum*) extracts, enol- to keto-transformation is the key factor in the synthesis of biogenic silver nanoparticles [79]. Sugars such as glucose and fructose exist in plant extracts can also be responsible for the formation of metallic nanoparticles. Note that glucose was capable of participating in the formation of metallic nanoparticles with different size and shapes, whereas fructose-mediated gold and silver nanoparticles are monodisperse in nature [80].

An FTIR analysis of green synthesized nanoparticles via plant extracts confirmed that nascent nanoparticles were repeatedly found to be associated with proteins [81]. Also, amino acids have different ways of reducing the metal ions. Gruen et al. [82] observed that amino acids (viz cysteine, arginine, lysine, and methionine are proficient in binding with silver ions. Tan et al. [83] tested all of the 20 natural α-amino acids to establish their efficient potential behavior towards the reduction of Au^0^ metal ions.

Plant extracts are made up of carbohydrates and proteins biomolecules, which act as a reducing agent to promote the formation of metallic nanoparticles [34]. Also, the proteins with functionalized amino groups (–NH_2_) available in plant extracts can actively participate in the reduction of metal ions [84]. The functional groups (such as –C–O–C–, –C–O–, –C=C–, and –C=O–) present in phytochemicals such as flavones, alkaloids, phenols, and anthracenes can help to generate metallic nanoparticles. According to Huang et al. [85], the absorption peaks of FTIR spectra at (1) 1042 and 1077, (2) 1606 and 1622, and (3) 1700–1800 cm^−1^ imply the stretching of (1) –C–O–C– or –C–O–, (2) –C=C– and (3) –C=O, respectively. Based on FTIR analysis, they confirmed that functional groups like –C–O–C–, –C–O–, –C=C–, and –C=O, are the capping ligands of the nanoparticles [86]. The main role of the capping ligands is to stabilize the nanoparticles to prevent further growth and agglomeration. Kesharwani et al. [87] covered photographic films using an emulsion of silver bromide. When light hit the film, the silver bromide was sensitized; this exposed film was placed into a solution of hydroquinone, which was further oxidized to quinone by the action of sensitized silver ion. The silver ion was reduced to silver metal, which remained in the emulsion.

Based on the chemistry of photography, we assumed that hydroquinone or plastohydroquinone or quinol (alcoholic compound) serve as a main reducing agent for the reduction of silver ions to silver nanoparticles through non-cyclic photophosphorylation [87]. Thus, this experiment proves that the biomolecules and heterocyclic compounds exist in plant extract were accountable for the extracellular synthesis of metallic nanoparticles by plants. It has already been well established that numerous plant phytochemicals including alkaloids, terpenoids, phenolic acids, sugars, polyphenols, and proteins play a significant role in the bioreduction of metal salt into metallic nanoparticles. For instance, Shanakr et al. [88] confirmed that the terpenoids present in geranium leaf extract actively take part in the conversion of silver ions into nanoparticles. Eugenol is a main terpenoid component of *Cinnamomum zeylanisum* (cinnamon) extracts, and it plays a crucial role for the bioreduction of HAuCl_4_ and AgNO_3_ metal salts into their respective metal nanoparticles. FTIR data showed that –OH groups originating from eugenol disappear during the formation of Au and Ag nanoparticles. After the formation of Au nanoparticles, carbonyl, alkenes, and chloride functional groups appeared. Several other groups [e.g., R–CH and –OH (aqueous)] were also found both before and after the production of Au nanoparticles [89]. Thus, they proposed the possible chemical mechanism shown in Fig. 3. Nonetheless, the exact fundamental mechanism for metal oxide nanoparticle preparation via plant extracts is still not fully tacit. In general, there are three phases of metallic nanoparticle synthesis from plant extracts: (1) the activation phase (bioreduction of metal ions/salts and nucleation process of the reduced metal ions), (2) the growth phase (spontaneous combination of tiny particles with greater ones) via a process acknowledged as Ostwald ripening, and (3) the last one is termination phase (defining the final shape of the nanoparticles) [90, 91]. The process of nanoparticle formation by plant extract is depicted in Fig. 4 [92].

**Fig. 3:** Schematic for the reduction of Au and Ag ions [89]

**Fig. 4:** Mechanism of nanoparticle formation by plant leaf extract [228]

## Environmental remediation applications

### Antimicrobial activity

Various studies have been carried out to ameliorate antimicrobial functions because of the growing microbial resistance towards common antiseptic and antibiotics. According to in vitro antimicrobial studies, the metallic nanoparticles effectively obstruct the several microbial species [93]. The antimicrobial effectiveness of the metallic nanoparticles depends upon two important parameters: (a) material employed for the synthesis of the nanoparticles and (b) their particle size. Over the time, microbial resistance to antimicrobial drugs has become gradually raised and is therefore a considerable threat to public health. For instance, antimicrobial drug resistant bacteria contain methicillin-resistant, sulfonamide-resistant, penicillin-resistant, and vancomycin-resistant properties [94]. Antibiotics face many current challenges such as combatting multidrug-resistant mutants and biofilms. The effectiveness of antibiotic is likely to decrease rapidly because of the drug resistance capabilities of microbes. Hence, even when bacteria are treated with large doses of antibiotics, diseases will persist in living beings. Biofilms are also an important way of providing multidrug resistance against heavy doses of antibiotics. Drug resistance occurs mainly in infectious diseases such as lung infection and gingivitis [95]. The most promising approach for abating or avoiding microbial drug resistance is the utilization of nanoparticles. Due to various mechanisms, metallic nanoparticles can preclude or overwhelm the multidrug-resistance and biofilm formation, as described in Figs. 5 and 6.

**Fig. 5:** Schematic for the multiple antimicrobial mechanisms in different metal nanoparticles against microbial cells [96]

**Fig. 6:** Various mechanisms of antimicrobial activity of metal nanoparticles [93]

Various nanoparticles employ multiple mechanisms concurrently to fight microbes [e.g., metal-containing nanoparticles, NO-releasing nanoparticles (NO NPs), and chitosan-containing nanoparticles (chitosan NPs)]. Nanoparticles can fight drug resistance because they operate using multiple mechanisms. Therefore, microbes must simultaneously have multiple gene mutations in their cell to overcome the nanoparticle mechanisms. However, simultaneous multiple biological gene mutations in the same cell are unlikely [96].

Multiple mechanisms observed in nanoparticles are discussed in Table 4. Silver nanoparticles are the most admired inorganic nanoparticles, and they are utilized as efficient antimicrobial, antifungal, antiviral, and anti-inflammatory agents [97]. According to a literature survey, the antimicrobial potential of silver nanoparticles can be described in the following ways: (1) denaturation of the bacterial outer membrane [98], (2) generation of pits/gaps in the bacterial cell membrane leading to fragmentation of the cell membrane [99, 100], and (3) interactions between Ag NPs and disulfide or sulfhydryl groups of enzymes disrupt metabolic processes; this step leads to cell death [101]. The shape-dependent antimicrobial activity was also examined. According to Pal et al. [102], truncated triangular nanoparticles are highly reactive in nature because their high-atom-density surfaces have enhanced antimicrobial activity.

**Table 4:** Multiple mechanisms of antimicrobial action for various metallic nanoparticles [96]

S. no.	Nanoparticles	Multiple mechanisms
1	Nitric oxide-releasing nanoparticles (NO NPs)	NO forms reactive nitrogen oxide intermediates (RNOS) by reacting with superoxide (O_2_^−^) (a) RNOS cause direct nitrosative damage to DNA, including causing strand breaks, formation of abasic sites and depleting the Fe in a bacterial cell (b) RNOS inactivate zinc metalloproteins, which results in inhibition of microbial cellular respiration (c) RNOS also cause lipid peroxidation
2	Chitosan-containing nanoparticles	(a) Due to its positive charge, chitosan binds with DNA in bacterial and fungal cells, thereby inhibiting transcription of mRNA resulting in protein translation (c) Chitosan also decreases the activities of metalloproteins
3	Silver-containing nanoparticles (Ag NPs)	The antimicrobial activity of silver (Ag) is due to its Ag^+^ ions (a) Ag^+^ inhibits the electron transport chain of microbes (b) Ag^+^ damages DNA and RNA by binding with them (c) Ag^+^ also inhibits cell division by inhibiting DNA replication (d) Ag^+^ ions form ROS, which are toxic to both bacterial cells and eukaryotic host cells
4	Zinc oxide-containing nanoparticles (ZnO NPs)	(a) ZnO NPs destroy both lipids and the proteins of the membrane, which can cause cell death (b) ZnO NPs also form Zn^2+^ ions and ROS, including hydrogen peroxide (H_2_O_2_),which damage the bacterial cell
5	Copper-containing nanoparticles	(a) Copper interacts with amine and carboxyl groups, which are present on microbes such as *B. subtilis* (b) Higher concentrations of Cu^2+^ ions can produce ROS
6	Titanium dioxide-containing nanoparticles (TiO_2_ NPs)	(a) In the photocatalysis process, TiO_2_ NPs generate ROS, including hydrogen peroxide (H_2_O_2_) and hydroxyl radicals (·OH), upon exposure to near-UV and UVA radiation
7	Magnesium-containing nanoparticles	(a) MgX_2_ NPs also cause lipid peroxidation of the microbial cell envelope by generating ROS (b) MgF_2_ NPs can cause lipid peroxidation and a drop in cytoplasmic pH, which raises membrane potential

The synthesis of Au nanoparticles is highly useful in the advancement of effective antibacterial agents because of their non-toxic nature, queer ability to be functionalized, polyvalent effects, and photo-thermal activity [103–105]. However, the antimicrobial action of gold nanoparticles is not associated with the production of any reactive oxygen species-related process [106]. To investigate the antibacterial potential of the Au nanoparticles, researchers attempted to attach nanoparticles to the bacterial membrane followed by modifying the membrane potential, which lowered the ATP level. This attachment also inhibited tRNA binding with the ribosome [106]. Azam et al. [107] examined the antimicrobial potential of zinc oxide (ZnO), copper oxide (CuO), and iron oxide (Fe_2_O_3_) nanoparticles toward gram-negative bacteria (*Escherichia coli*, *Pseudomonas aeruginosa*) and gram-positive bacteria (*Staphylococcus Aureus* and *Bacillus subtilis*). Accordingly, the most intense antibacterial activity was reported for the ZnO nanoparticles. In contrast, Fe_2_O_3_ nanoparticles exhibited the weakest antibacterial effects. The order of antibacterial activities of nanoparticles was found to be as ZnO (19.89 ± 1.43 nm), CuO (29.11 ± 1.61 nm), and Fe_2_O_3_ (35.16 ± 1.47 nm). These results clearly depicts that the size of the nanoparticles also play a momentous role in the antibacterial potential of each sample [107]. The anticipated mechanism of antimicrobial action of ZnO nanoparticles is: (1) ROS generation, (2) zinc ion release on the surface, (3) membrane dysfunction, and (4) entry into the cell. Also, the antimicrobial potential of ZnO nanoparticles is concentration and surface area dependent [108]. Mahapatra et al. [109] determined the antimicrobial action of copper oxide nanoparticles towards several bacterial species such as *Klebsiella pneumoniae*, *P. aeruginosa*, *Shigella Salmonella paratyphi* s. They found that CuO nanoparticles exhibited suitable antibacterial activity against those bacteria. It was assumed that nanoparticles should cross the bacterial cell membrane to damage the crucial enzymes of bacteria, which further induce cell death. For instance, green synthesized nanoparticles show enhanced antimicrobial activity compared to chemically synthesized or commercial nanoparticles. This is because the plants [such as *Ocimum sanctum* (Tulsi) and *Azadirachta indica* (neem)] employed for synthesis of nanoparticles have medicinal properties [110, 111]. For example, green synthesized silver nanoparticles showed an efficient and large zone of clearance against various bacterial strains compared to commercial silver nanoparticles (Fig. 7) [112].

**Fig. 7:** Schematic for the antimicrobial activity for the five bacterial strains: **a** *Staphylococcus aureus*, **b** *Klebsiella pneumonia*, **c** *Pseudomonas aeruginosa*, **d** *Vibrio cholera*, and **e** *Proteus vulgaris*. Numbers of 1 through 6 inside each strain denote: (1) nickel chloride, (2) control ciprofloxacin, (3) *Desmodium gangeticum* root extract, (4) negative control, (5) nickel NPs prepared by a green method, and (6) nickel NPs prepared by a chemical method [229]

### Catalytic activity

4-Nitrophenol and its derivatives are used to manufacture herbicides, insecticides, and synthetic dyestuffs, and they can significantly damage the ecosystem as common organic pollutants of wastewater. Due to its toxic and inhibitory nature, 4-nitrophenol is a great environmental concern. Therefore, the reduction of these pollutants is crucial. The 4-nitrophenol reduction product, 4-aminophenol, has been applied in diverse fields as an intermediate for paracetamol, sulfur dyes, rubber antioxidants, preparation of black/white film developers, corrosion inhibitors, and precursors in antipyretic and analgesic drugs [113, 114]. The simplest and most effective way to reduce 4-nitrophenol is to introduce NaBH_4_ as a reductant and a metal catalyst such as Au NPs [115], Ag NPs [116], CuO NPs [117], and Pd NPs [118]. Metal NPs exhibit admirable catalytic potential because of the high rate of surface adsorption ability and high surface area to volume ratio. Nevertheless, the viability of the reaction declines as a consequence of the substantial potential difference between donor (H_3_BO_3_/NaBH_4_) and acceptor molecules (nitrophenolate ion), which accounts for the higher activation energy barrier.

Metallic NPs can promote the rate of reaction by increasing the adsorption of reactants on their surface, thereby diminishing activation energy barriers [119, 120] (Fig. 8). The UV–visible spectrum of 4-nitrophenol was characterized by a sharp band at 400 nm as a nitrophenolate ion was produced in the presence of NaOH. The addition of Ag NPs (synthesized by *Chenopodium aristatum* L. stem extract) to the reaction medium led to a fast decay in the absorption intensity at 400 nm, which was concurrently accompanied by the appearance of a comparatively wide band at 313 nm, demonstrating the formation of 4-aminophenol [121] (Fig. 9).

**Fig. 8:** Schematic of the metallic NP-mediated catalytic reduction of 4-nitrophenol to 4-aminophenol [120]

**Fig. 9:** UV-visible spectra illustrating *Chenopodium aristatum* L. stem extract synthesized Ag NP-mediated catalytic reduction of 4-NP to 4-AP at three different temperatures **a** 30 °C, **b** 50 °C, and **c** 70 °C. Reduction in the absorption intensity of the characteristic nitrophenolate band at 400 nm accompanied by concomitant appearance of a wider absorption band at 313 nm indicates the formation of 4-AP [121]

### Removal of pollutant dyes

Cationic and anionic dyes are a main class of organic pollutants used in various applications [122]. Organic dyes play a very imperative role due to their gigantic demand in paper mills, textiles, plastic, leather, food, printing, and pharmaceuticals industries. In textile industries, about 60% of dyes are consumed in the manufacturing process of pigmentation for many fabrics [123]. After the fabric process, nearly 15% of dyes are wasted and are discharged into the hydrosphere, and they represent a significant source of pollution due to their recalcitrance nature [124]. The pollutants from these manufacturing units are the most important sources of ecological pollution. They produce undesirable turbidity in the water, which will reduce sunlight penetration, and this leads to the resistance of photochemical synthesis and biological attacks to aquatic and marine life [125–127]. Therefore, the management of effluents containing dyes is one of the daunting challenge in the field of environmental chemistry [128].

The need for hygienic and safe drinking water is increasing day by day. Considering this fact, the use of metal and metal oxide semiconductor nanomaterials for oxidizing toxic pollutants has become of great interest in recent material research fields [129–131]. In the nano regime, semiconductor nanomaterials have superior photocatalytic activity relative to the bulk materials. Metal oxide semiconductor nanoparticles (like ZnO, TiO_2_, SnO_2_, WO_3_, and CuO) have been applied preferentially for the photocatalytic activity of synthetic dyes [31, 132–134]. The merits of these nanophotocatalysts (e.g., ZnO and TiO_2_ nanoparticles) are ascribable to their high surface area to mass ratio to enhance the adsorption of organic pollutants. The surface energy of the nanoparticles increases due to the large number of surface reactive sites available on the nanoparticle surfaces. This leads to an increase in rate of contaminant removal at low concentrations. Consequently, a lower quantity of nanocatalyst will be required to treat polluted water relative to the bulk material [135–138]. Like metal oxide nanoparticles, metal nanoparticles also show enhanced photocatalytic degradation of various pollutant dyes; for example, silver nanoparticles synthesized from *Z. armatum* leaf extract were utilized for the degradation of various pollutant dyes [127] (Fig. 10).

**Fig. 10:** Schematic for the reduction of **a** safranine O, **b** methyl red, **c** methyl orange, and **d** methylene blue dyes using silver NPs synthesized from *Z. armatum* leaf extract by metallic nanoparticles [136]

### Heavy metal ion sensing

Heavy metals (like Ni, Cu, Fe, Cr, Zn, Co, Cd, Pb, Cr, Hg, and Mn) are well-known for being pollutants in air, soil, and water. There are innumerable sources of heavy metal pollution such as mining waste, vehicle emissions, natural gas, paper, plastic, coal, and dye industries [139]. Some metals (like lead, copper, cadmium, and mercury ions) shows enhanced toxicity potential even at trace ppm levels [140, 141]. Therefore, the identification of toxic metals in the biological and aquatic environment has become a vital need for proper remedial processes [142–144]. Conventional techniques based on instrumental systems generally offer excellent sensitivity in multi-element analysis. However, experimental set ups to perform such analysis are highly expensive, time-consuming, skill-dependent, and non-portable.

Due to the tunable size and distance-dependent optical properties of metallic nanoparticles, they have been preferably employed for the detection of heavy metal ions in polluted water systems [145, 146]. The advantages of using metal NPs as colorimetric sensors for heavy metal ions in environmental systems/samples include simplicity, cost effectiveness, and high sensitivity at sub ppm levels. Karthiga et al. [147] synthesized AgNPs using various plant extracts used as colorimetric sensors for heavy metal ions like cadmium, chromium, mercury, calcium, and zinc (Cd^2+^, Cr^3+^, Hg^2+^, Ca^2+^, and Zn^2+^) in water. Their as-synthesized Ag nanoparticles showed colorimetric sensing of zinc and mercury ions (Zn^2+^ and Hg^2+^). Likewise, AgNPs synthesized using mango fresh leaves and dried leaves (fresh, MF-AgNPs and sun-dried, MD-AgNPs) exhibited selective sensing for mercury and lead ions (Hg^2+^ and Pb^2+^). Also, AgNPs prepared from pepper seed extract and green tea extract (GT-AgNPs) showed selective sensing properties for Hg^2+^, Pb^2+^, and Zn^2+^ ions [147] (Fig. 11).

**Fig. 11:** Schematic of metal removal using metal oxides prepared by green synthesis. Left—**a** digital images and **b** absorption spectra of neem bark extract-mediated silver NPs (NB-AgNPs) with different metal ions and concentration-dependent studies of **c** Hg^2+^ and **d** Zn^2+^. Right—**a** digital images and **b** absorption spectra of fresh mango leaf extract-mediated silver NPs (MF-AgNPs) with different metal ions and **c** concentration-dependent studies of Pb^2+^ removal [147]

## Conclusion and future prospects

‘Green’ synthesis of metal and metal oxide nanoparticles has been a highly attractive research area over the last decade. Numerous kinds of natural extracts (i.e., biocomponents like plant, bacteria, fungi, yeast, and plant extract) have been employed as efficient resources for the synthesis and/or fabrication of materials. Among them, plant extract has been proven to possess high efficiency as stabilizing and reducing agents for the synthesis of controlled materials (i.e., controlled shapes, sizes, structures, and other specific features). This review article was organized to encompass the ‘state of the art’ research on the ‘green’ synthesis of metal/metal oxide nanoparticles and their use in environmental remediation applications. Detailed synthesis mechanisms and an updated literature study on the role of solvents in synthesis have been reviewed thoroughly based on the literature available to help encounter the existing problems in ‘green’ synthesis. In summary, future research and development of prospective ‘green’ materials/nanoparticle synthesis should be directed toward extending laboratory-based work to an industrial scale by considering traditional/present issues, especially health and environmental effects. Nevertheless, ‘green’ material/nanoparticle synthesis based on biocomponent-derived materials/nanoparticles is likely to be applied extensively both in the field of environmental remediation and in other important areas like pharmaceutical, food, and cosmetic industries. Biosynthesis of metals and their oxide materials/nanoparticles using marine algae and marine plants is an area that remains largely unexplored. Accordingly, ample possibilities remain for the exploration of new green preparatory strategies based on biogenic synthesis.
